# Research on Forest Conversation Analysis Using Autoregressive Neural Network-Based Model

**DOI:** 10.1155/2022/3280928

**Published:** 2022-06-20

**Authors:** Tianhao Ma, Yuchen She, Junang Liu

**Affiliations:** ^1^College of Forestry, Central South University of Forestry and Technology, Changsha, 410004 Hunan, China; ^2^Central South Inventory and Planning Institute of National Forestry and Grassland Administration, Changsha, 410014 Hunan, China

## Abstract

Forest biodiversity is an important component of biological diversity that should not be disregarded. The question of how to evaluate it has sparked scholarly inquiry and discussion. The purpose of this paper is to describe the principles of general linear regression, the selection of model variables in OLS autoregressive modelling, model coefficient testing, analysis of variance of autoregressive models, and model evaluation indicators in order to clarify the suitability of GWR models for solving biomass-related data problems. The GWR 4.0 program was used to create a spatially weighted autoregressive model. Model testing and an accuracy analysis were performed on the model. Following a comparison and study with the general linear regression model, it was discovered that the geographically weighted autoregressive model is better suited to defining spatially correlated data than the general linear regression model.

## 1. Introduction

Since the industrial revolution, the impact of human activities on the biosphere has spread from local to global, especially the concentration of *CO*_2_, *CH*_4_ and other greenhouse gases in the atmosphere is increasing year by year, resulting in a continuous increase in global temperature [1]. The rise in global temperature will lead to a rise in sea level, an uneven distribution of precipitation, increased desertification and natural disasters, which will seriously affect the development of national economies [2].

Forest biomass is the carrier of the carbon cycle in forest ecosystems and an important parameter for assessing the forest carbon cycle [3]. There are basically three traditional ways to study forest biomass: firstly, the micrometeorological field method, which combines the rules of micrometeorological field with wind direction, wind speed and temperature; secondly, the carbon dioxide balance method, which measures the change of carbon dioxide in the ecosystem; and thirdly, the direct harvesting method, which investigates the existing biomass of the forest, although this method is more accurate, it is difficult to use because of the large workload, complicated process and long period; Accurate determination of forest biomass is important for both production and theoretical research, and has been valued by ecologists and foresters worldwide [4]. The use of forest biomass models to estimate biomass has become a popular method.

There are three basic types of forest biomass models: linear models, non-linear models and polynomial models. These models are based on the basic assumption that the biomass distribution is random and do not take into account the spatial non-stationarity of the study variables [5]. It has been found that the spatial correlation between many sample data is due to the proximity of geographical locations; in order to take into account the spatial correlation of data when studying biomass distribution, In recent years, the evaluation of forest biodiversity has been studied more from a systemic perspective, and the factors affecting the evaluation include not only natural factors, but also various factors such as human, social and economic development [6]. The methods proposed to prevent the decline of biodiversity include not only natural measures, but also socio-economic and cultural measures. For example, concluded that the decline of species and biological assets is mainly caused by the neglect of ecological values other than private interests, and proposed that ecosystems and biodiversity the scientific assessment process for ecosystems and biodiversity is policy change [7]. Studies by [8, 9] also show that habitat loss and habitat fragmentation are major contributors to environmental degradation and biodiversity loss. In addition, it is difficult to know the exact number of species, ecosystems and genes in forest biodiversity, no matter how it is evaluated, and its evaluation is a typical ‘black box' system [10]. The evaluation of forest biodiversity is a typical “black box” system, and the “black box” theory should be applied to evaluate changes in forest biodiversity through the pressure-state and response caused by human socio-economic activities [11]. The author takes the biodiversity of forest nature reserves as the research object, collects relevant information based on the data of the seven national forest resources inventories, and establishes a differential equation between biodiversity changes and economic development in forest nature reserves at the national level to find out the optimal price for forest biodiversity value evaluation, with a view to providing a basis for biodiversity value compensation and management [12].

The paper's organization paragraph is as follows: The related work is presented in Section 2.  Section 3 analyzes the geographically weighted regression of the proposed work.  Section 4, discusses the comparative analysis of results. Finally, in Section 5, the research work is concluded.

## 2. Related Work

In a study of the application of geographically weighted autoregressive models, [13] for the first time used a geographically weighted regression model to study the distribution of disease and compared it with the traditional least squares method, showing that the residuals of the method were much smaller than those of the ordinary linear regression model. [14] Established a spatial relationship between China's GDP and the variation of each province. The usual regression analysis assumes that the regression coefficients are consistent across regions, but in actual geographical space, the impact of a certain factor on the level of industrialization development is not entirely consistent across regions. This method is a good way to analyses the relationship between the local economy and the overall economy and the process of change. [In Sendai, Japan, he studied the spatial variation of the heat island effect in the city and showed that the same spatial variation in urban temperature trends could be addressed by a geographically weighted autoregressive model. [15] Used the geographically weighted autoregressive principle to model the relationship between climate and elevation in the UK, and showed that the model fit was very well matched to reality. [16] used a GWR model to successfully solve the spatial distribution pattern of vegetation. In the same year, [17, 18] applied this method to the analysis of regional industrialisation and his results showed that the level of industrialisation varied significantly spatially due to environmental influences. [8] applied this method to traffic, studying the relationship between average visual traffic and environmental factors, and thus predicting future traffic congestion levels in different regions [19].

In general, a lot of research has been done in geographically weighted regression at home and abroad, and a lot of results have been achieved. However, forest biomass distribution research is limited to classic geostatistical approaches and remote sensing spectral analysis, which leaves a lot to be desired. Geographically weighted regression models have great advantages in solving the spatial distribution of geographic things, especially the new geographically weighted regression models, whose powerful function type is getting more and more attention and application [19]. Therefore, the geographically weighted regression models used in this paper simulate the spatial distribution of forest biomass, and it is important to analyze the advantages and disadvantages of geographically weighted regression models in the spatial distribution of forest biomass [20–22].

## 3. Geographically Weighted Regression

In forest manager surveys, the distribution characteristics of all the data we collect often vary depending on location. Traditional regression analysis methods ignore the relationship between parameter estimates and the geographical location of data collection and fail to represent the spatial sub-characteristics of the data. To address this problem.

### 3.1. Geographically Weighted Regression Model Basis

It has the following basic form:

(1) $$\begin{array}{c} y_{i}=\beta_{0}\left(u_{i},v_{i}\right)+\overset{p}{\underset{k=1}{\sum }}\beta_{k}\left(u_{i},v_{i}\right)x_{ik}+\varepsilon_{i}\;i=1,2\cdots ,n \end{array}$$

Where (*u*_*i*_, *v*_*i*_) is the geographical coordinate of the ith sampling point, *β*_*k*_(*u*_*i*_, *v*_*i*_) is the kth regression coefficient on the ith sampling point, *ε*_*i*_ is the random error term, and the underlying assumption is that it follows a normal distribution, i.e.

(2) $$\begin{array}{c} \varepsilon_{i}\sim N\left(0,\sigma^{2}\right)\text{Cov}\left(\varepsilon_{i},\varepsilon_{j}\right)=0\left(i\neq j\right) \end{array}$$

Equation (2) can also be written as:

(3) $$\begin{array}{c} y_{i}=\beta_{i0}+\overset{p}{\underset{k=1}{\sum }}\beta_{ik}x_{ik}+\varepsilon_{i}\;i=1,2\cdots ,n \end{array}$$

If *β*_1*k*_ = *β*_2*k*_ = ⋯ = *β*_*nk*_, then the GWmin model is the same as the general linear regression model, i.e, which will W better reflect the spatial variation patterns of the study variables. To simplify the calculation process, Brunsdon et al. introduced a spatial weight *w*_*ij*_ into the model so that the regression parameters at point i would have to make

(4) $$\begin{array}{c} \overset{n}{\underset{j=1}{\sum }}w_{ij}{\left(y_{j}-\beta_{i0}-\overset{p}{\underset{k=1}{\sum }}\beta_{ik}x_{ik}\right)}^{2} \end{array}$$

The estimated value of the regression parameter is calculated when the minimum value is taken as $\hat{\beta }\left(u_{i},v_{i}\right)$, where *w*_*ij*_ is the geographical weight, the size of which increases as the geographical distance between point i and point j decreases.

The estimated value of the regression parameter $\hat{\beta }\left(u_{i},v_{i}\right)$ at observation point i is:

(5) $$\begin{array}{c} \hat{\beta }\left(u_{i},v_{i}\right)={\left(X^{\prime }W\left(u_{i},v_{i}\right)X\right)}^{-1}X^{\prime }W\left(u_{i},v_{i}\right)Y \end{array}$$

Of which:

(6) $$\begin{array}{c} X=\left[\begin{array}{cccc} 1 & x_{11} & \cdots & x_{1k}\\ 1 & x_{21} & \cdots & x_{2k}\\ \cdots & \cdots & \cdots & \cdots \\ 1 & x_{n1} & \cdots & x_{nk} \end{array}\right],W\left(u_{i},v_{i}\right)=W_{i}=\left[\begin{array}{cccc} w_{i1} & 0 & \cdots & 0\\ \cdots & w_{i2} & \cdots & 0\\ \cdots & \cdots & \cdots & \cdots \\ 0 & 0 & \cdots & w_{\text{in}} \end{array}\right] \end{array}$$

(7) $$\begin{array}{c} \beta =\left[\begin{array}{cccc} \beta_{0}\left(u_{1},v_{1}\right) & \beta_{1}\left(u_{1},v_{1}\right) & \cdots & \beta_{k}\left(u_{1},v_{1}\right)\\ \beta_{0}\left(u_{2},v_{2}\right) & \beta_{1}\left(u_{2},v_{2}\right) & \cdots & \beta_{k}\left(u_{2},v_{2}\right)\\ \cdots & \cdots & \cdots & \cdots \\ \beta_{0}\left(u_{n},v_{n}\right) & \beta_{1}\left(u_{n},v_{n}\right) & \cdots & \beta_{k}\left(u_{n},v_{n}\right) \end{array}\right],Y=\left[\begin{array}{c} y_{1}\\ y_{2}\\ \cdots \\ y_{n} \end{array}\right] \end{array}$$

n is the number of sample sites, $\overset{⌢}{\beta }$ is the estimated value of the regression coefficient slice, and k is the number of independent variables. *w*_*ij*_(*j* = 1, 2, ⋯, *n*) is the weight given to sample point j when fitting the model at observation i.

*X*_*i*_ is the vector consisting of the ith observed independent variable factor, and according to Equation (7), the fitted value ${\hat{y}}_{i}$ is obtained as

(8) $$\begin{array}{c} {\hat{y}}_{i}=X_{i}\hat{\beta }\left(u_{i},v_{i}\right)=X_{i}{\left(X^{\prime }W\left(u_{i},v_{i}\right)X\right)}^{-1}X^{\prime }W\left(u_{i},v_{i}\right)Y \end{array}$$

The matrix shape of the fitted values can be expressed as follows:

(9) $$\begin{array}{c} \hat{Y}=\left[\begin{array}{c} X_{1}{\left(X^{\prime }W\left(u_{1},v_{1}\right)X\right)}^{-1}X^{\prime }W\left(u_{1},v_{1}\right)\\ X_{2}{\left(X^{\prime }W\left(u_{2},v_{2}\right)X\right)}^{-1}X^{\prime }W\left(u_{2},v_{2}\right)\\ \cdots \\ X_{n}{\left(X^{\prime }W\left(u_{n},v_{n}\right)X\right)}^{-1}X^{\prime }W\left(u_{n},v_{n}\right) \end{array}\right]Y=SY \end{array}$$

Where

(10) $$\begin{array}{c} \text{S}=\left[\begin{array}{c} X_{1}{\left(X^{\prime }W\left(u_{1},v_{1}\right)X\right)}^{-1}X^{\prime }W\left(u_{1},v_{1}\right)\\ X_{2}{\left(XW\left(u_{2},v_{2}\right)X\right)}^{-1}XW\left(u_{2},v_{2}\right)\\ \cdots \\ X_{n}{\left(X^{\prime }W\left(u_{n},v_{n}\right)X\right)}^{-1}X^{\prime }W\left(u_{n},v_{n}\right) \end{array}\right] \end{array}$$

is the spatial hat matrix of the geographically weighted back coincidence fit.

### 3.2. Selection of Spatial Enumeration Functions

The spatial weights are used to represent the degree of relationship prior to the regression point's neighboring point j. Equation Equation (9) provides the definition of spatial weights, which is used to calculate the GWR model's regression parameters. The following four spatial weight functions are commonly used, respectively.

#### 3.2.1. Distance Threshold Method

Distance threshold method is actually given a distance D, such as is less than the distance D is considered to be the weight of 1, otherwise the weight is considered to be 0, that is, the points beyond the distance is considered irrelevant to the current point, the distance outside the point does not participate in the model fitting calculation. The formula is expressed as follows:

(11) $$\begin{array}{c} w_{ij}=\left\{\begin{array}{cc} 1 & d_{ij}\leq D\\ 0 & d_{ij}>D \end{array}\right. \end{array}$$

#### 3.2.2. The Inverse Distance Method

The inverse distance method was proposed by the scholar Tobler and the formula is expressed as follows:

(12) $$\begin{array}{c} w_{ij}=1/d_{ij}^{\alpha } \end{array}$$

Where is a constant that is determined by the situation. The formula above shows that the closer the point is to the center, the more weight it receives. Tobler proposed it mostly based on the first law of geography. The inverse distance method is much better than the distance threshold, but the only drawback is that if the regression points overlap with the sample data points *d*_*ij*_^*α*^ = 0, then the weights appear to be infinite at this point. If this point is removed, the accuracy of the parameter estimation is reduced, so this method is also not applicable to GWR models.

(13) $$\begin{array}{c} w_{ij}=\exp\left(-{\left(d_{ij}/b\right)}^{2}\right) \end{array}$$

Where b is the bandwidth. From the formula, the larger the bandwidth, the slower the decay of the weights, and vice versa. If b =0, then *w*_*ij*_ = 1, which means that the weight at regression point i is 1 and the weights at other observation points tend to be 0, the fit becomes a local fit. If b is infinite, then the weights at all observation points converge to 1, and the fit is in fact a global fit. If the bandwidth is fixed, the *w*_*ij*_ = 1 weights reach a maximum when *d*_*ij*_ = 0; *w*_*ij*_ decreases as the distance between the sample point and the regression point increases.

#### 3.2.3. Truncated Function Method (Bi-Square)

Gaussian function will be the sample data involved in the calculation, while the truncated function only calculates the distance less than the bandwidth of the sample data, truncated function is to improve the efficiency of the calculation of Gaussian function of the improved type, the form of the following:

(14) $$\begin{array}{c} w_{ij}=\left\{\begin{array}{cc} \left[{\left[1-{\left(d_{ij}/b\right)}^{2}\right]}^{2}\right. & d_{ij}\leq b\\ 0 & d_{ij}>b \end{array}\right. \end{array}$$

### 3.3. Geographically Weighted Regression Model Implementation Method

In this paper, the geo-weighted regression model was calculated using GWR4.0, a Gaussian kernel function was used for the fitting process, and C V was used as the evaluation index to select the best bandwidth. The dependent variable of the model was the forest biomass of each sample plot, the environmental factor Elevation and the average diameter at breast height (AVER DBH) of the stand were used as independent variables. The GWR model was expressed as follows: the biomass *y*_*i*_ per hectare of sample plot number i was expressed as the sum of the product of the jth independent variable *x*_*ij*_(j = 0, 1, 2) and the corresponding coefficient (*β*_*ij*_, *j* = 0, 1, 2), and *ε* was the model residual.

(15) $$\begin{array}{c} y_{i}=\beta_{i0}+\beta_{i1}x_{i1}+\beta_{i2}x_{i2} \end{array}$$

Where *y*_*i*_ is the biomass per hectare in plot i, *x*_*i*1_ is the elevation of plot i, *x*_*i*2_ is the mean diameter at breast height in plot i and *ε* is the model residual.

A weighting function is used in the GWR model to quantify the effect of each site biomass on the forest biomass of the sample site. The weight function chosen in this paper is a Gaussian function with a bandwidth of 1083 m and the weight function is shown below:

(16) $$\begin{array}{c} w_{ij}=e^{-{\left(\frac{d_{ij}}{1083}\right)}^{2}} \end{array}$$

## 4. Comparative Analysis of Results

The five evaluation indicators for the two models are given in Table 1. From the table, it can be seen that the AIC value of the GWR model is 18.325 smaller than the ALC value of the OLS model. In addition, the AICc and CV of the local model are much smaller than those of the traditional linear regression model, which further indicates that the local model has improved the accuracy of biomass estimation, and that the R2 and R2-squared values have increased further compared to those of the OLS model. Because the geographically weighted regression model handles spatial unsteadiness in its modelling, these measures suggest that the GwR model's model accuracy, predictive power, and precision are substantially higher than those of the OLS model.

The estimated values, standard errors, p-values, *β*-1 × SD and *β* +1 × SD of the least squares model coefficients are shown in Table 2. For the general linear regression model, the model coefficients showed significant correlation at the a =0.05 level of significance.

In terms of model coefficients, mean diameter at breast height was the most important factor. Another important factor is elevation. The data show that forest biomass is higher at higher elevations and lower at lower elevations. Lower elevations are flatter and more heavily damaged by humans, but higher elevations have steeper slopes and are less prone to tree removal, resulting in larger forest biomass. The GWwR model is a local regression model in which a set of local regression parameters is calculated for each regression point, and the variation between the regression parameters can explain the spatial non-stationarity of the predictors very well. The spatial non-stationarity of the study factors can be well explained by the variation between regression parameters. The results of the geographically weighted regressions for the Liangshui National Nature Reserve include: maximum, minimum, median, 25% quantile (Q1) and 75% quantile (Q3). As shown in Table 3.

National studies have found that the median GWR model coefficient is similar to the OLS model coefficient; between Q1 (25% quantile) and Q3 (75% quantile) 50% of the GwR model coefficients are included. If the data meet the basic assumption of a normal distribution, with 68% of the OS model coefficients included within ±1 standard deviation of the model coefficients, it is generally accepted that if there is no non-stationarity in the spatial distribution of the data, then the geo-weighted regression model coefficients Q1 and Q3 should be included within ±1 standard deviation of the least squares model coefficients. If Q1 or Q3 do not fall within the range [*β*-1 × SDB+1xSD], then there is non-stationarity in the spatial distribution of the study variables. 1 For example, the range of Q1 to Q3 for the coefficients of the AVER DBH values in the geo-weighted regression is 5.04 to 7.7 [22–25].

This demonstrates the spatial non-stationarity of the relationship between the mean diameter at breast height and the elevation coefficients. With the development of GIS technology, the spatial variation of the coefficients of the geo-weighted regression model can be visualised using GIS technology to produce maps. Figures 1 and 2 use maps to depict the spatial distribution patterns of these regression coefficients. The mean diameter at breast height of the sample plots is generally positive throughout the study area, whereas elevation varies from negative to positive in different areas.

The scatter plots of the residuals of the GWR model and the OLS model are shown in Figures 3 and 4, respectively. This indicates that the GWR model is more accurate and solves the heteroskedasticity problem to a certain extent.

Local residuals spatial correlation analysis Global Moran'sI can only reflect the spatial correlation of the study variables as a whole. The local Moran'sI statistic was introduced in this research to further investigate the spatial correlation of model residuals in different regions. In order to make comparative analysis easier, a bandwidth of 1083 m was selected and the local Moran'sI statistic of the residuals was calculated using the EXCEL plug-in ROOTCASE, and finally the Moran'sI was plotted using the bubble chart tool in EXCEL. The results are shown in Figure 5.

## 5. Conclusions

The fundamentals of general linear auto regression, model variable selection in OLS regression modelling, model coefficient tests, regression model analysis of variance, and model evaluation indicators are all covered in this work. The weighting function selection procedure in the geographically weighted regression model is presented, as well as the pros and disadvantages of each weighting function, and the Gaussian function is finally chosen as the weighting function in this study. The selection methods and criteria of different bandwidths are presented, and after comparison, the model finally decides to choose 1083 m as the bandwidth to achieve forest value protection.

## Figures and Tables

**Figure 1:** Spatial distribution of regression coefficients.

**Figure 2:** Spatial distribution of elevation regression coefficients.

**Figure 3:** GWR residual distribution.

**Figure 4:** OLS Residuals Distribution Chart.

**Figure 5:** OLS residual local spatial correlation.

**Table 1:** Two model fit statistics.

Model	AIC	AICc	*R* ^2^	*R*_*adj*_^2^	CV
OLS	1324.741	1223.147	0.554	0.521	2164.010
GWR	1305.421	1254.291	0.745	0.654	1954.623

**Table 2:** Linear back old model coefficients, standard errors and *p*-values.

Variable	Estimate	StandardError	T value	Pr > t	*β*-1 × SD	*β*+1 × SD
Intercept	-54.021	23.412	-2.010	0.0214	-75.241	-31.247
Elevation	0.157	0.0640	2.630	0.008	0.099	0.214
AVER_DBH	6.321	0.5620	11.24	<0.001	5.741	6.852

**Table 3:** Estimated values of the 3GTO model parameters.

Variable	Mean	Standard	Min	Lwr quartile	Median	Upr quartile	Max
Intercept	-32.14	76.54	-214.75	-74.40	-74.23	1.15	189.61
Elevation	0.09	0.23	-0.35	-0.480	0.07	0.25	0.60
AVER_DBH	6.50	1.47	0.23	5.240	7.01	7.80	10.54

## Data Availability

The datasets used during the current study are available from the corresponding author on reasonable request.
